The article "Prevalence and Motives of Social Media Use among the Iranian Population" was published in 2022. Journal: J Environ Public Health.

# Prevalence and Motives of Social Media Use among the Iranian Population

**DOI:** 10.1155/2022/1490227

**Published:** 2022-04-01

**Authors:** Maryam Chegeni, Nouzar Nakhaee, Mahin Eslami Shahrbabaki, Parvin Mangolian Shahrbabaki, Sara Javadi, AliAkbar Haghdoost

**Affiliations:** ^1^Department of Basic and Medical Laboratory Sciences, Khomein University of Medical Sciences, Khomein, Iran; ^2^Molecular and Medicine Research Center, Khomein University of Medical Sciences, Khomein, Iran; ^3^Health Services Management Research Center, Institute for Futures Studies in Health, Kerman University of Medical Sciences, Kerman, Iran; ^4^Neuroscience Research Center, Institute of Neuropharmacology, Department of Psychiatry, Kerman University of Medical Sciences, Kerman, Iran; ^5^Department of Critical Care Nursing, Kerman University of Medical Sciences, Kerman, Iran; ^6^Kerman University of Medical Sciences, Kerman, Iran; ^7^HIV/STI Surveillance Research Center, and WHO Collaborating Center for HIV Surveillance, Institute for Futures Studies in Health, Kerman University of Medical Sciences, Kerman, Iran

## Abstract

**Background:**

Around the world, people are using social media (SM) for different purposes following a wide range of patterns. There is a paucity of studies addressing the issue in the Eastern Mediterranean region. In this population-based study, the frequency and patterns of SM use in Iran were investigated.

**Materials and Methods:**

To explore the prevalence and motives of SM use, a sample of 1800 Iranian people aged 10–65 years old (53.5% female) were surveyed. Social media addiction (SMA) was assessed using the Bergen Social Media Addiction Scale.

**Results:**

The results revealed that 88.5% (*n* = 1593) of the participants were SM users, and the average time spent by them in SM was 4.0 ± 3.9 hours. The most common motivations for SM use were communication with others (48.9%), receiving news (40.7%), and surfing the net (40.6%). Besides, burning eyes (31.0%), headache (26.8%), and sleep disturbance (25.1%) were the most common health problems experienced by SM users. The SMA prevalence was 23.1% (95% CI: 21.2, 25.1) (males: 23.8%; females: 22.5%), with a higher rate (26.0%) among adolescents and young people.

**Conclusion:**

SM use and SMA appear to be real health challenges in Iran, particularly among youth. Consequently, to decrease the negative impacts of excessive SM use, exploring the motives behind SM use and designing population-based interventions are recommended.

## 1. Introduction

Social media (SM) including WhatsApp, Instagram, and Facebook have been considerably affecting people's daily lives. Users often tend to develop their virtual social life on a SM platform. According to the latest statistics, an estimated 3.6 billion people were using SM worldwide in 2020, a number that is predicted to increase to almost 4.41 billion in 2025 [1]. The average time spent in SM by Internet users worldwide in 2019 was estimated to be 144 minutes per day compared to 142 minutes in the previous year [2]. Recent data from Financial Tribune [3] reflected approximately 47 million people (57% of the population) who can be marked as active SM users in Iran, representing an 18% increase in the year before.

The article "Prevalence and Motives of Social Media Use among the Iranian Population" was published in 2022. Journal: J Environ Public Health.

Unfortunately, excessive use of SM has been a common problem affecting the majority of the total population of users. They have developed an interest in using SM while working, eating with family members, and even walking in the street [4]. Furthermore, SM and communication technologies strongly influence the decision-making process of users, in relation to health communication, especially to particular health issues currently much discussed (e.g., consciously choosing to adhere to vaccination schedules) [5]. SM users spend a considerable amount of time communicating with friends and reading the materials posted by other members while being unaware of adverse effects of problematic usage [6].

Moreover, the excessive use of SM could cause psychological [7], physical [8, 9], and emotional difficulties [10, 11], dysfunction [11, 12], social and work problems [13], and induce personal and family conflicts for users [14]. Excessive and impulsive use of SM can be considered social media addiction (henceforth SMA) [15]. We intend to evaluate SM addiction before the COVID-19 pandemic, but it is so important to pay attention to SM addiction during the pandemic. Recently, the literature has examined the effect of social isolation caused by COVID-19 on SM addiction [16].

Therefore, identifying the motivations that lead people to excessive use of SM is essential. Studies have found various motivations such as communication with family [17], complement or compensate for low social status [18], entertainment, chatting, social networking, and surfing the net [19] as factors underlying SM use. Besides, a study in Kuwait as a country in the Eastern Mediterranean Region (EMRO) pointed to entertainment, information seeking, personal utility, and convenience as motivations for using SM [20].

However, so far, there is no estimate of the SMA prevalence in the general population in EMRO, especially in Iran. To fill the research gap, this study explores the prevalence of SM use, SMA, motivations that attract people to SM, and physical health problems caused by SM in Iranian general population.

## 2. Materials and Methods

### 2.1. Participants and Setting

The present study was conducted in Kerman, a city located in the southeast of Iran. The province has a population of 3.4 million as the largest province of Iran, and 85.4% of the population is literate [19].

The article "Prevalence and Motives of Social Media Use among the Iranian Population" was published in 2022. Journal: J Environ Public Health.

Visitors to hospitals of Kerman constituted the sampling frame in this study. Our previous experience suggests that this sampling frame is a fair representative sample of total population [21]. The sample consisted of 1800 persons aged 10–65 years. To this end, companions of patients who had been referred to private and public hospitals in Kerman to visit patients were included in the research sample. It should be noted the participants were not patients. We used self-administered questions instead of interviews. Questioners had been waited for participants to complete the questionnaires, and there was no specific time limit.

The data were collected anonymously, and the sealed ballot box method was applied to ensure confidentiality of the participants' information.

### 2.2. Measures

The questionnaire consisted of the following parts.

### 2.3. Social Media Addiction

SMA was assessed using the Bergen Social Media Addiction Scale (BSMAS) [22]. BSMAS is a six-item self-report tool used to assess six core components including salience, mood modification, tolerance, withdrawal, conflict, and relapse [23]. The scale adapted previously in the Iranian population showed good validity and reliability properties in the Persian language [24]. In our study, Cronbach's alpha was 0.72.

### 2.4. Questions Related to SM

#### 2.4.1. Motives for SM Use

The questions related to the motivation to use SM were adapted from a qualitative study conducted in Iran [24]. An expert panel confirmed the content validity of it. The main question was “Why do you usually use social media?” People could choose more than one option and write to us if they had a reason other than the one mentioned. It consisted of 13 items. Items such as communicating with others, receiving news, surfing, entertainment, learning, escaping from loneliness, forgetting problems, attractiveness of social media, finding new friends, work, meeting emotional needs, excitement-seeking, and competition. Each item was measured with a yes or no scale, and finally, the frequency of items was measured.

Meanwhile, to identify the type of SM platform use, a question was embedded as “Which social media do you use?” People could choose more than one option, and if they are users of another SM whose name was not in the options, write it to us. This list included WhatsApp, Telegram, Instagram, Facebook, Twitter, YouTube, Iranian platforms (such as Soroush and Gap), Line, Viber, and Emo.

The article "Prevalence and Motives of Social Media Use among the Iranian Population" was published in 2022. Journal: J Environ Public Health.

#### 2.4.2. Health Problems Associated with SM Use

The questions related to the health problems associated with SM use were adapted from a qualitative study conducted in Iran [24]. The main question was “ Have you ever had any of the following health problems due to using social media?” People could choose more than one option, and if they had any health problems related to using SM but were not in the options, write to us. These problems included headache, eye problems (burning eyes and eye pain), musculoskeletal problems (arm, neck, wrist pain, and tingling of fingers), and sleep disturbance.

### 2.5. Demographics

This study addresses demographic and family characteristics such as age, gender, level of education, job, family size, marital status, years of marriage, and residence (in rural and urban areas).

### 2.6. Statistical Analysis

Unadjusted and multivariate-adjusted logistic regression analyses were performed to find out if there is any association between SMA and demographic variables. Besides, to determine if SMA (the response variable) has any relationship with other research variables, the unadjusted logistic model was used. Thereafter, all variables with a *p* value of less than 0.2 were included in the adjusted logistic model. Eventually, the final model was developed using the backward method. All statistical procedures were performed using STATA 16 software at a significance level of 0.05 (*α* < 0.05).

### 2.7. Ethics

This study was approved by the ethics committee (IR.KMU.REC.1397.338). According to the requirements of the university's ethics committee, verbal consent was obtained from the participants before entering into the study.

## 3. Results

The response rate in this study was 97.2% (1750 out of 1800 participants), and the participants were aged 10–65 years (*M* = 27.1, SD = 10.3). The female participants accounted for 53.5% of the total sample (*n* = 964). In the current study, 88.5% (*n* = 1593) of the participants were SM users, and their average daily usage was 4.0 ± 3.9 hours.

The most frequently used SM were WhatsApp (68.4%), Telegram (65.7%), and Instagram (61.1%), respectively (Figure 1).

As given in Table 1, the SMA prevalence on average was 23.1% (95% CI: 21.2, 25.1) with the highest rate among adolescents (26.3%) (95% CI: 22.7, 30.2) followed by young people (26.2%) (95% CI: 23.3, 29.2).

There were significant differences between the two groups of SM addicts and normal users in terms of the age, marital status, and place of residence (Table 2).

The most common motivations for people to use SM were communication with others (48.9%, 95% CI: 46.6, 51.2), receiving news (40.7%, 95% CI: 38.4, 43.0), and surfing the net (40.6%, 95% CI: 38.3, 42.9) (Figure 2).

The article "Prevalence and Motives of Social Media Use among the Iranian Population" was published in 2022. Journal: J Environ Public Health.

Burning eyes (31.0%, 95% CI: 28.9, 33.2), headache (26.8%, 95% CI, 24.8, 28.9), and sleep disturbances (25.1%, 95% CI: 23.1, 27.1) were the most common physical health problems experienced by the SM users (Figure 3).

## 4. Discussion

This study aimed to assess the prevalence, motives, and correlates of SM use among Iranian population.

Overall, 88.5% of 10–65-year-old people in southeastern Iran were SM users, and the most common SM platforms used by them were WhatsApp, Telegram, and Instagram. WhatsApp is also the most popular platform among Finns, while in other countries such as Philippines, Sweden, and Norway, Facebook and YouTube are the most commonly used platforms [2].

According our results, SM users spend an average of 4.0 hours (240 minutes) in SM platforms each day. This is a substantial figure almost resembling the time spent in SM by the Philippines. Based on the latest online usage statistics, in 2019, SM users in the Philippines were ranked first as they spent over 4 hours per day using SM [2]. In comparison, the daily time spent with SM in the U.S was just 116 minutes [2], which is half the daily time spent in Iran. However, most of this time is spent by Iranians for communicating with others and entertainment.

This time spent in SM is important because it has a positive relationship with SMA [25].

In this study, 23.1% of the participants were affected by SMA. Wartberg [26], Bányai [27], and Mérelle [28] reported a problematic SM use prevalence of 2.6%, 4.5%, and 9.1% for a representative sample of German, Hungarian, and Dutch adolescents, while we observed a SMA prevalence estimate of 26.0% in Iranian adolescents and young adults. However, some studies have reported a higher prevalence rate than the rate reported in the present study, e.g., the prevalence of 47% in Malaysian college students [29], 44% in U.S. young adults [30], and approximately 40% among Bangladeshi students [31]. In addition to cultural factors, these differences can be attributed to various methodological issues such as the use of convenience sampling, focusing mainly on college students, having small sample sizes, and variations in diagnostic criteria and assessment tools used for diagnosis.

The present study found that age, marital status, and place of residence were significantly associated with SMA. However, the observed SMA associations with education, job, family size, year of marriage, and gender were not significant in the final adjusted model.

In short, the findings of these studies demonstrated that the participants who were single, young, and resident in rural areas tended to report higher scores on the SMA scale.

The article "Prevalence and Motives of Social Media Use among the Iranian Population" was published in 2022. Journal: J Environ Public Health.

According to our findings, the prevalence of SMA among Iranian adolescents and young people was two times greater than the rate reported by people over 35 years of age. The results of the present study are in line with many studies conducted worldwide. For instance, some studies have suggested that younger people are more attached to SM and are more likely to be addicted to them than other age groups [26, 32, 33]. However, it has been shown that these users are more likely to suffer from complications such as decreased mental health [34], loss of positive emotions [11], poor sleep quality [33], declined academic performance [20, 33], psychological and wellbeing disorders [35, 36], loneliness [10], depression, and anxiety [7] due to excessive use of SM. Furthermore, given that the age composition of Iran is young, a large number of people are at the risk of negative consequences of excessive SM use.

Following previous studies in the literature, the present study found that single people including unmarried people, widows, and divorced people were more affected by addictive use of SM than married people [37, 38]. Given the higher frequency of SM use for communication with others and entertainment, it can be assumed that single people have more time and are more willing to communicate with others through these networks.

According to this study, living in cities seems to decrease the chances of addiction to SM. However, Pawłowska [39] reported that adolescents living in urban areas showed a significantly greater interest in using the Internet compared to those living in rural areas. Some studies showed that there is no significant difference between the prevalence of Internet addiction in rural and urban areas [40, 41]. Overall, it seems that access to welfare amenities and diverse entertainment facilities can help to spend less time on SM. However, considering these differences, it seems that more studies are needed to investigate the effect of the place of residence on SMA especially in Iran.

It seems important to know the reasons for this high presence of SM use. Approximately, one out of three people stated that their motivation was to be on SM to communicate with others, receive news, surfing the net, and entertain. In general, competition, excitement-seeking, and meeting emotional needs were the least frequently cited motivating factors for using SM.

A study showed that college students living in Kuwait used SM mainly for entertainment, information seeking, personal utility, and convenience [20]. However, it was shown that entertainment motivation increases compulsive SM use (YouTube) [42], an issue that needs to be confirmed by further studies.

The article "Prevalence and Motives of Social Media Use among the Iranian Population" was published in 2022. Journal: J Environ Public Health.

This study indicated that the most common health problems due to the use of SM were burning eyes (31.0%), headache (26.8%), and sleep disturbance (25.1%). Sleep disturbance has been reported in other studies such as in Bengaluru 26.1% [43] and US young adults 57.0% [44]. Other studies have also suggested associations between SM use and sleep disturbance in countries such as Australia and China [45, 46]. A recent review in this area demonstrated an inverse association between electronic media use and sleep parameters such as longer time to fall asleep, delayed bedtime, and reduced total sleep time [47]. Increased anxiety levels have been widely shown as one of the most important factors leading to sleep deprivation [48]. Another study suggested that sleep deprivation can result in mood deficits such as depression, anger, confusion, anxiety, vigor, and fatigue [49]. Moreover, among musculoskeletal problems, neck pain (21.4%) was found as the most common problem among the participants. In line with our study, neck and upper back complaints had the highest prevalence rates ranging from 55.8% to 89.9% [9].

A major limitation of the present study was that the cross-sectional nature of the data limited our ability to establish directionality. There was a possibility of response-related biases, since the data were collected using self-report instruments. Despite these limitations, the target population in this study was representative of the general population covering various age groups living in southeast Iran. This study contributed to the literature on the SMA prevalence and the associated factors. However, further studies are necessary for proper assessment of SMA in Iran. On the other hand, early awareness is important for policymakers to examine the problems associated with SM use and implement effective measures to prevent them.

Since, in this study, the data collection process was completed before December 2019, we could not examine the impact of the epidemic on social media addiction. It is recommended to evaluate the prevalence of SM use, SMA, motivations that attract people to SM, and physical health problems caused by SM considering the social isolation caused by the COVID-19 epidemic. The results of our study and their comparison with related studies in the postepidemic period can lead to valuable results in relation to SM addiction.

## Figures and Tables

**Figure 1:** Social media platforms used by the participants (*N*  = 1800).

**Figure 2:** Motives of social media use among Iranian community (*N*  = 1800).

**Figure 3:** The prevalence of complications caused by social media use among Iranian community (*N*  = 1800).

The article "Prevalence and Motives of Social Media Use among the Iranian Population" was published in 2022. Journal: J Environ Public Health.

**Table 1:** The participants' characteristics by social media addiction.

		SMA (%)	*P* value
Gender	Male	196 (23.8)	0.52
	Female	216 (22.5)	
Age	≤18 y	143 (26.3)	<0.001
	18–35 y	224 (26.2)	
	>35 y	45 (11.7)	
Job	Housewife or retired	85 (18.2)	<0.001
	Employee (in public or private sectors)	146 (22.2)	
	Student	172 (28.3)	
Level of education	Academic education	154 (22.7)	0.77
	Diploma	120 (22.6)	
	High school and lower education	138 (24.3)	
Marital status	Single	258 (28.0)	<0.001
	Married	159 (18.2)	
Family size	Mean ± SD	4.3 ± 1.53	0.14
Residence	Urban area	351 (22.4)	
	Rural area	57 (29.0)	0.03

**Table 2:** Odds ratio (95% CI) for social media addiction in the final model of logistic regression.

Adjusted model		
Age	>35 y	Reference
	18–35 y	2.25 (1.57, 3.23) < 0.001
	18 y	1.88 (1.21, 2.90) 0.004
Marital status	Married	Reference
	Single	1.51 (1.14, 2.01) 0.004
Residence	Urban area	Reference
	Rural area	1.41 (1.01, 1.97) 0.043

Adjusted by level of education, job, residence, family size, year of marriage, and marital status.

## Data Availability

The data used to support the findings of this study are available by sending the email to the authors.
